# Transcriptomic Profile Analysis of *Streptococcus mutans* Response to *Acmella paniculata* Flower Extracts

**DOI:** 10.1155/2022/7767940

**Published:** 2022-06-21

**Authors:** Siti Aisyah Abd Ghafar, Nur Syahirah Salehuddin, Nor Zaihana Abdul Rahman, Nadia Halib, Rohazila Mohamad Hanafiah

**Affiliations:** Department of Basic Science and Oral Biology, Faculty of Dentistry, Universiti Sains Islam Malaysia, Kuala Lumpur 55100, Malaysia

## Abstract

**Background:**

*Acmella paniculata* has been used as a traditional medicine to treat oral health diseases such as dental caries and periodontitis. *Streptococcus mutans* is a common bacterium that initiates dental caries at an early stage.

**Aim:**

The aim of this study was to determine the mode of action of *A*. *paniculata* (extracts) against *S*. *mutans* growth.

**Methods:**

Time-kill assay has been done to investigate the rate of kill and effectiveness of *Acmella paniculata* (AP) extracts against *S*. *mutans* growth. Phytochemical analysis was done to identify major compounds in AP extracts using gas chromatography mass spectrometry (GCMS). Scanning and transmission electron microscopy (SEM and TEM) have been done to observe the morphological changes of treated bacteria. Transcriptomic profile analysis has been done using Next Gene Sequencing.

**Results:**

AP flower n-hexane (APFH) and AP flower dichloromethane (APFD) extracts acted as bactericidal agents after killing >3 log10 cfu/mL of *S. mutans* after 24 hours. Oleic and hexadecenoic acids were found to be the major compounds in APFD and APFH extracts, respectively. Photomicrographs from SEM and TEM of treated *S*. *mutans* show that the bacterial cell wall has been lysed and the cytoplasm content was decreased. Pathway analysis revealed that the APFD extract significantly affected biosynthesis peptidoglycan, gene expression, RNA processing, and macromolecule metabolism processes in *S*. *mutans*.

**Conclusion:**

Data analysis revealed that multiple mechanisms of action were involved in antibacterial activity of *A*. *paniculata* extracts toward *S*. *mutans*.

## 1. Introduction

Dental caries, also known as tooth decay or cavities, has become a common disease worldwide and is generally experienced by children. It is a process that involves the balance between mineral loss and replacement in the teeth in a certain period of time, as the reaction effect of acid attack resulting from food intake. Dental caries incident is affected by the frequency and amount of carbohydrate from starch and sugar that were consumed. *Streptococcus mutans* is a common bacterium that initiates dental caries at an early stage. This bacterium is able to convert sugar into acid and form plaque on teeth. This situation is becoming extremely challenging as commonly used antibiotics and chemotherapeutics such as penicillin, cephalosporin, erythromycin, and tetracycline have begun to be less effective against oral bacteria [1]. In addition, Prestinaci et al. (2015) stated that prolonged exposure to antibiotic drugs can cause major safety issues, for example, the development of resistant microorganisms [2]. Therefore, they will have a greater chance of surviving and multiplying. Furthermore, mouthrinse consumption may cause oral cancer due to its alcohol content, particularly in smokers and/or those who consume alcohol on a regular basis [3]. In addition, the use of mouthrinse has also been linked to the occurrence of enamel staining and the formation of calculus, which has limited its usage as oral hygiene preventive measures [4]. Therefore, many researchers have begun to find a new alternative by developing safer and organic medicines that offer effective plaque control with no or at least minimal side effects.

Bioactive compounds from plant extraction have been found to be effective as anti-microorganism, antidepressant, and antidiabetic agents with less minimal side effects [5–7]. Some examples of medicinal plants that have potential to be anti-microorganism agents are *Andrographis paniculata*, *Lepidagathis hyalina*, *Syzygium fruticosum*, and green tea [8–11]. They contain bioactive compounds responsible for inhibiting the growth of bacteria and viruses such as lactones, diterpenes, flavonoids, quinic acid, xanthones, and noriridoids.

Spilanthes acmella, an attractive medicinal plant, and its metabolites have the potential to be antibacterial agents. It is also a synonym species for *Acmella paniculata* and has been used as a traditional medicine for many diseases such as rheumatism, fever, diuretics, flu, toothaches, and periodontitis. Previous studies have stated that this plant exhibits analgesic, cytotoxic, antimicrobial, and antiplaque effects [12]. Phytochemicals present in *Acmella* species such as alkyl ketones, alkamides, hydrocarbons, acetylenes, lactones, alkaloids, terpenoids, flavonoids, and coumarins are the main constituents considered to be responsible for the anti-microorganism activity [13–15]. Besides, toxicity level of *A*. *paniculata* extract was found to be the lowest and safe for animal. According to Dubey et al., crude extract of A*. paniculata* can be used in animal feed at 0.01% v/v and 1% v/v, respectively, without any lethal, sublethal, or malformation effect [16].

Even though *A. paniculata* is believed traditionally to be an anti-toothache plant, scientific proof of the mechanism of action on the biological activity has yet to be reported. Therefore, the aim of this study was to investigate the mode of action of bioactive compounds from *A. paniculata* against *S. mutans* using an antimicrobial assay and transcriptomic profile analysis.

## 2. Materials and Methods

### 2.1. Sample Extraction

*Acmella paniculata* (AP) was collected at TKC Herbal Ampangan, Seremban. The plant was identified by Dr. Mohd Firdaus Ismail, a botanist from Institute of Bioscience, Universiti Putra Malaysia (UPM) (Voucher number: MF10164120). The extraction has been done by following the method from Nur Syahirah et al. [17]. The leaves of AP have been extracted using n-hexane and methanol solvents, whereas the flowers of AP have been extracted using n-hexane and dichloromethane (DCM) solvents.

### 2.2. Bacterial Growth

*Streptococcus mutans* (ATCC 25175) was cultured in brain heart infusion broth (BHIB) for 24 hours under facultative anaerobic condition. Then, the culture was grown on brain heart infusion agar (BHIA) to obtain a single colony. The single colony was further investigated in this study.

### 2.3. Time-Kill Assay

*Streptococcus mutans* (ATCC 25175) was cultured in Mueller–Hinton broth (MHB) (Oxoid) at 37°C for 24 hours under facultative anaerobic condition. Dilution had been done on overnight culture at 0.5 cfu/mL. About 200 *µ*L of culture was transferred into 20 mL of MHB with (12.5–100 mg/mL) *A. paniculata* leaves n-hexane (APLH), *A. paniculata* leaves methanol (APLM), *A. paniculata* flower n-hexane (APFH), and *A. paniculata* flower dichloromethane (APFD) extracts. All the samples were incubated at 37°C for 24 hours under facultative anaerobic conditions. Samples (100 *µ*L) were then cultured on tryptic soy agar (TSA) at 0, 4, 8, 24, and 28 hours. Killing curves were constructed by plotting the log_10_ cfu/mL versus time over 24 hours.

### 2.4. Scanning Electron Microscopy (SEM)

*S*. *mutans* was cultured on Mueller–Hinton agar (MHA) at 37°C under facultative anaerobic conditions with MIC and MBC values of 12.5 and 50 mg/mL for both APFH and APFD extracts, respectively. Control was prepared as an untreated culture. Each sample was incubated for 4 hours. After incubation, the agar was cut into 1 cm × 1 cm × 1 cm (square cm^3^). All the samples were transferred into a 1.5 mL Eppendorf tube. Fixation of the samples was done by treating them with glutaraldehyde 2% for 24 hours at 4°C. After that, all the samples were washed using PBS 0.1 M. Then, a drying process was done on all the samples using ethanol and critical point under CO_2_ conditions. The samples were then placed on stubs and covered with gold before being observed using a scanning electron microscope (Carl Zeiss LEO 1450VP).

### 2.5. Transmission Electron Microscopy (TEM)

*S. mutans* was cultured on brain heart infusion broth (BHIB) (0.5 × 108 cfu/mL) with MIC and MBC values of 12.5 and 50 mg/mL for both APFN and APFD extracts at 37°C under facultative anaerobic conditions. The BHIB contained 0.2% sucrose. Control had been prepared as an untreated culture. The time of incubation was four hours for each sample. After that, 10 mL of culture was centrifuged at 4000 rpm and 4°C for 15 minutes. The pellet was collected and washed with PBS 0.1 M. Glutaraldehyde 2% had been added to samples for 24 hours at 4°C. Then, fixation was done by adding osmium tetroxide for 2 hours. Then, a drying process was done on all the samples using ethanol (50–90%). The samples had been embedded in epoxy resin. After that, uranyl acetate and Reynolds' stain were added to the samples. The samples had been cut into thin ultrathin slices before being observed using a transmission electron microscope (Philips CM12).

### 2.6. Gas Chromatography Mass Spectrophotometry (GCMS) Analysis

Bioactive compounds from APFH and APFD extracts were determined by GCMS analysis (Shimadzu, QP5050 A, Japan). Helium gas (1.0 mL/min) was used as a carrier gas in this analysis. The temperature and time for the setting were set at 60°C in 2 minutes and 280°C in 12 minutes, respectively. After that, the injector was maintained at 245°C, while the electron impact of the ion source was maintained at 295°C. Electron impact spectra were logged at 70 eV. The bioactive compounds were determined by comparing the GC retention indices with the mass spectra library provided by the National Institute of Standards and Technology (NIST) database.

### 2.7. RNA Extraction

Two pellets of treated bacteria (APFD 1 × MIC) and untreated bacteria were prepared for RNA extraction. All the samples were suspended in 3.2 mL of SDS lysis buffer and divided into four portions. Each portion (∼800 *μ*L) was transferred into a 2 mL tube containing bead; 100 *μ*L of phenol : chloroform : isoamyl alcohol; and 100 *μ*L of enhanced lysis buffer. The cells were lysed by bead beating for 5 min at 2280 rpm on a cell disruptor. The sample tubes were then centrifuged for 2 min at full speed. The supernatants were pooled into a 15 mL tube to a final volume of 2.5 mL. Aliquots of 313 *μ*L of binding buffer were added, vortexed, and incubated for 2 min at room temperature. The tube was then centrifuged for 2 min at full speed. The supernatant was transferred into a column (including a filter) which was pre-equilibrated with 12 mL of equilibration buffer. The filter column was flushed and washed with washing buffers. RNA was then eluted with 5 mL of elution buffer. The first eluted RNA was mixed with 3.5 mL of isopropanol, loaded into a purification column, and centrifuged for 2 min at full speed. The column was washed with buffer followed by drying using centrifugation force for 2 min at full speed. Finally, the RNA was eluted with 100 *μ*L of water. The RNA sample was subjected to DNase treatment at 37°C, followed by column purification and concentration. Lastly, the purified RNA was dissolved in 40 *μ*L of water. RNA degradation and contamination were monitored on 1% agarose gels. RNA purity was checked using a NanoPhotometer® spectrophotometer (IMPLEN, CA, USA). RNA integrity and quantitation were assessed using the RNA 6000 Nano Assay Kit of the Bioanalyzer 2100 system (Agilent Technologies, CA, USA).

### 2.8. Transcriptomic Profile of Treated Bacteria

#### 2.8.1. Library Preparation for Transcriptome Sequencing

A total of 1 *μ*g RNA per sample was used as input material for the RNA sample preparations. Sequencing libraries were generated using NEBNext® Ultra™ RNA Library Prep Kit for Illumina® (NEB, USA) following manufacturer's recommendations, and index codes were added to attribute sequences to each sample. Briefly, mRNA was purified from total RNA using poly-T oligo-attached magnetic beads. Fragmentation was carried out using divalent cations under elevated temperature in NEBNext First Strand Synthesis Reaction Buffer (5X). First strand cDNA was synthesized using random hexamer primer and M-MuLV Reverse Transcriptase (RNase H−). Second strand cDNA synthesis was subsequently performed using DNA polymerase I and RNase H. Remaining overhangs were converted into blunt ends via exonuclease/polymerase activities. After adenylation of 32032 ends of DNA fragments, NEBNext adaptor with hairpin loop structure was ligated to prepare for hybridization. In order to select cDNA fragments of preferentially 150∼200 bp in length, the library fragments were purified with AMPure XP system (Beckman Coulter, Beverly, USA). Then, 3 *μ*L USER Enzyme (NEB, USA) was used with size-selected, adaptor-ligated cDNA at 37°C for 15 min followed by 5 min at 95°C before PCR. Then, PCR was performed with Phusion High-Fidelity DNA polymerase, Universal PCR Primers, and Index (*X*) Primer. Lastly, PCR products were purified (AMPure XP system), and library quality was assessed on the Agilent Bioanalyzer 2100 system.

#### 2.8.2. Clustering and Sequencing

The clustering of the index-coded samples was performed on a cBot Cluster Generation System using PE Cluster Kit cBot-HS (Illumina) according to the manufacturer's instructions. After cluster generation, the library preparations were sequenced on an Illumina platform, and paired-end reads were generated.

#### 2.8.3. Quality Control

Raw data (raw reads) of FASTQ format were firstly processed through fastp. In this step, clean data (clean reads) were obtained by trimming reads containing adapter and removing poly-N sequences and reads with low quality from raw data. At the same time, Q20, Q30, and GC content of the clean data were calculated. All the downstream analyses were based on the clean data with high quality.

#### 2.8.4. Reads Mapping to the Reference Genome

Reference genome and gene model annotation files were downloaded from genome website directly. Both building index of reference genome and aligning clean reads to reference genome were conducted using Bowtie 2 [18].

#### 2.8.5. Quantification of Gene Expression Level

featureCounts was used to count the reads' numbers mapped to each gene. Then, FPKM of each gene was calculated based on the length of the gene and reads' count mapped to this gene. FPKM, expected number of fragments per kilobase of transcript sequence per million base pairs sequenced, considers the effect of sequencing depth and gene length for the read count at the same time and is currently the most commonly used method for estimating gene expression levels [19].

#### 2.8.6. Differential Expression Analysis

For DESeq2 with biological replicates, differential expression analysis of two conditions/groups (two biological replicates per condition) was performed using the DESeq2 R package. DESeq2 provides statistical routines for determining differential expression in digital gene expression data using a model based on the negative binomial distribution. The resulting *p* values were adjusted using the Benjamini and Hochberg's approach for controlling the false discovery rate. Genes with adjusted *p* value <0.05 found by DESeq2 were assigned as differentially expressed.

#### 2.8.7. GO and KEGG Enrichment Analysis of Differentially Expressed Genes

Gene ontology (GO) enrichment analysis of differentially expressed genes was implemented by the clusterProfiler *R* package, in which gene length bias was corrected. GO terms with corrected *p* value less than 0.05 were considered significantly enriched by differential expressed genes. KEGG is a database resource for understanding high-level functions and utilities of the biological system, such as the cell, the organism, and the ecosystem, from molecular level information, especially large-scale molecular datasets generated by genome sequencing and other high-throughput experimental technologies https://www.genome.jp/kegg/. ClusterProfiler *R* package was used to test the statistical enrichment of differential expression genes in KEGG pathways.

## 3. Results

### 3.1. Time-Kill Assay

The results presented in the time-kill assay are the changes in the log_10_ cfu/mL of viable colonies. Bactericidal activity was defined as reduction equal to or greater than 3 log_10_ cfu/mL in the viable colony count relative to the initial inoculum [20]. Time-kill assay was performed using MIC and MBC concentration values from previous study for APLH, APLM, APFH, and APHD extracts [17]. MIC and MBC values for APLH and APLM extracts were 25 mg/mL and 100 mg/mL, respectively. Meanwhile, the MIC and MBC values for APFH and APFD extracts were 12.5 mg/mL and 50 mg/mL, respectively. The finding of time-kill assay is presented in Table 1. After 4-hour incubation, *S*. *mutans* treated with APLM, APLH, APFH, and APFD extracts (MIC) was reduced by a range of 0.91–2.07 log_10_ cfu/mL. After 8 hours of incubation, the log reduction in the viable cell count ranged between 0.84 and 2.17 log_10_ cfu/mL. Log reduction equal to or greater than 3 log_10_ cfu/mL occurred when cells were treated with 2 × MIC APLM, APLH, APFH, and APFD extracts from 4 until 8 hours of incubation, respectively. Obvious reduction of *S*. *mutans* (log_10_ cfu/mL) has been observed when it is treated with 1 × MIC APFH and APFD extracts.

### 3.2. SEM Analysis

Scanning electron microscopy (SEM) and transmission electron microscopy (TEM) analysis were carried out to unravel *S*. *mutans* morphology after being exposed to APFD and APFH extracts for 4 h. SEM and TEM analysis were focused only on APFD and APFH because they exhibit greater antibacterial activities when compared to APLM and APLH. SEM analysis showed that the morphology of untreated *S*. *mutans* (control group) was aggregated preferentially within clusters (Figure 1(a)). Morphology of *S*. *mutans* exposed to APFH at 12.5 mg/mL and 50 mg/mL was changed when compared to control (Figures 1(b) and 1(c)). The close-up micrographs of the same culture showed that *S*. *mutans* cells became elongated and shrunk. A few holes were found on the surface of *S*. *mutans* cells, and smaller size of *S*. *mutans* cells was observed because of leakage from cytoplasm content. *S*. *mutans* treated with APFD at 12.5 mg/mL and 50 mg/mL was observed to have lysed, wrinkled cell walls and a lack of cytoplasm content (Figures 1(d) and 1(e)).

### 3.3. TEM Analysis

TEM analysis results showed untreated *S*. *mutans* (control) presence with bodies, granules, vacuoles, and cell membrane that encapsulated the bacterial cells (Figure 2(a)). On the other hand, TEM images of *S*. *mutans* treated with APFD extracts (12.5 and 50 mg/mL) showed lysis of the cell wall and decreased cytoplasm content (Figures 2(b) and 2(c)). Disintegration of membrane cells due to cytoplasm leakage represents an abnormal intracellular reaction of treated bacteria. The coccus shape of *S*. *mutans* was not conserved and distorted after being treated with APFH extracts at 12.5 and 50 mg/mL (Figures 2(d) and 2(e)). The morphological characteristics of treated cells were observed as the presence of changes in peripheral cell surface and formation of hollows, and cells were destroyed.

### 3.4. GCMS Analysis

GCMS analysis was carried out to identify bioactive compounds in APFH and APFD extracts. The bioactive compounds of APFD and APFH extracts are given in Tables 2 and 3, respectively. The ion chromatograms of APFD and APFH extracts are given in Figures 3 and 4, respectively. The peaks in the chromatogram were integrated and compared with the database of spectra of known components from the GCMS library. The volatile compounds with the highest peaks in APFD extract were linoelaidic acid, octadecanoic acid, and palmitoleic acid. Meanwhile, the highest peaks of bioactive compounds in APFH extract were hexadecanoic acid and oleic acid. Phytochemical analysis of APFD and APFH extracts revealed the presence of different fatty acids and heterocyclic compounds.

### 3.5. Transcriptomic Profile Analysis

#### 3.5.1. RNA Extraction Analysis

Transcriptomic profile analysis has been done to determine the differential expression genes (DEGs) of *S*. *mutans* treated with APFD (MIC) extract for 4 hours. APFD extract was used for this analysis because it exhibited greater antibacterial activity in SEM and TEM analysis compared with APFH extract. Four RNAs were successfully extracted from two treated bacteria (1 × MIC APFD) and two untreated bacteria (Control). The concentration and RNA integrity number (RIN) analysis for all samples are given in Table 4. The RNA integrity numbers of all samples were more than 8.6. The RNA samples were further utilized to investigate the gene expression profile of treated *S*. *mutans*.

#### 3.5.2. Mapping to Reference Genome

The genome of SmuNN2025 has been used as a reference genome when mapping against untreated and treated *S*. *mutans* RNA. The result of the mapping was more than 90% for all the samples. The highest genome mapping score was the control sample, above 95% (Table 5). The accuracy of genome mapping analysis should be more than 70%, and the percentage of mapping to multiple sites in the reference genome should be less than 10%.

#### 3.5.3. Gene Expression Level

Gene expression levels were measured by transcript abundance. The greater the transcript abundance, the higher the gene expression level. The gene expression level is estimated by counting the reads mapped to genes or exons. The number of reads is proportionate not only to the level of gene expression, but also to the gene length and the sequencing depth. In order for the gene expression levels estimated from different genes and experiments to be comparable, the number of fragments per kilobase of transcript sequence per million base pairs sequenced (FPKM) was used. In RNA-sequence, FPKM is the most common method of estimating gene expression levels, which takes into account the effects of both sequencing depth and gene length on the counting of fragments [19]. featureCounts software was used to analyze the gene expression levels in this experiment. The result files present the number of genes with different expression levels and the expression level of single genes. In general, FPKM value of 0.1 or 1 was set as the threshold for determining whether the gene is expressed or not. The comparison of treated and untreated genes has been done using duplicate samples. RNA-sequence analysis showed that APFD extract has significant (*p* < 0.05) effects on the transcriptomic profile of *S*. *mutans* compared to control. Out of 1266 genes, 622 genes were downregulated, and 644 genes were upregulated (Figure 5). Data analysis of differential expression genes (DEGs) showed that APFD extracts strongly induced the differential expression (11, *p* < 0.05). Gene expression changes were visualized as a heatmap and volcano plot to identify specific genes with high fold changes and statistical significance. The results of the heatmap and volcano plot are shown in Figures 6(a) and 6(b). Genes that were significantly different are expressed and presented in red (upregulated) and blue (downregulated).

#### 3.5.4. Upregulated and Downregulated Genes

In APFD-treated S. *mutans*, genes of biosynthesis peptidoglycan such as *murD*, *uppS*, *murC2*, *pbp2b*, *murE*, *murN*, and *murB* were among the top downregulated genes. All the genes are responsible for forming peptidoglycan in *S. mutans*.  Table 6 contains a list of downregulated genes involved in peptidoglycan biosynthesis. Other genes that were also strongly downregulated when treated with APFD were DNA replication genes such as *SmuNN2025_1359*, *ssb*, *dnaG*, *rnh3*, and *holB*.

The genes that were strongly upregulated when treated with APFD (MIC) were those encoding proteins involved in microbial metabolism in diverse environments, such as *pdhD*, *pf1*, *pdhA*, *SmuNN2025_1677*, *glk*, Ldh and *serA*. Genes that were upregulated during treatment are frequently involved in the bacterial response to other environmental stress conditions like heat exposure, osmotic shock, or starvation conditions [21]. A list of upregulated genes is given in Table 7.

#### 3.5.5. Gene Ontology Enrichment Analysis

Further investigation has been done to investigate the biological functions and the metabolic pathway by analyzing the gene ontology (GO) of *S*. *mutans* treated with APFD extract. The GO categories of DEGs are shown in Figure 7. It is divided into three sections: molecular function, cellular components, and biological processes. GO terms with padj <0.05 were regard as significant enrichment. In molecular function (MF), about 20 categories were downregulated, and nucleic acid binding of molecular function was higher compared to other categories (Figure 7(a)). Meanwhile, genes involved in the binding process were the most downregulated after being treated with APFD. In cellular components, about 19 of cell components were downregulated after *S*. *mutans* was treated with APFD (Figure 7(b)). The cytoplasmic component was the most downregulated after being treated with APFD. About 524 genes of cellular components were downregulated in this analysis. Gene expression, RNA processing, and macromolecular metabolic processes were the most enriched biology process for downregulated DEGs in the presence of APFD (Figure 7(c)). The most downregulated genes were involved in the biological process and cellular component.

#### 3.5.6. KEGG Enrichment Analysis

The interactions of multiple genes may be involved in certain biological functions. KEGG (Kyoto Encyclopedia of Genes and Genomes) is a collection of manually curated databases dealing with genomes, biological pathways, diseases, drugs, and chemical substances. KEGG is utilized for bioinformatics research and education, including data analysis in genomics, metagenomics, metabolomics, and other omics studies. Pathway enrichment analysis identifies significantly enriched metabolic pathways or signal transduction pathways associated with differentially expressed genes compared with the whole genome background.  Figure 8 is a KEGG enrichment scatter plot of DEGs (downregulated) for *S*. *mutans* treated with APFD extract. The extract induced differential expression of genes (downregulated) involved in the ribosome, DNA replication, peptidoglycan biosynthesis, and bacterial secretion system of *S*. *mutans*.

## 4. Discussion

This study was a continuation of previous research which investigated the antibacterial activities of *A*. *paniculata* extracts against *S*. *mutans* [17]. From previous studies, the minimum inhibitory concentration of APLH and APLM was 25 mg/mL, and that of APFH and APFD was 12.5 mg/mL. Meanwhile, the minimum bactericidal concentrations of the samples were 50 mg/mL for APLH, APFD, and APFH. However, MBC value for APLM was 100 mg/mL. This study was furthered by investigating the rate of kill and the effectiveness of the sample bactericidal activity as indicated by the time-kill assay. Bactericidal activity is achieved when the extracts reduce >3 log_10_ colony forming units (cfu) from the initial inoculum. Meanwhile, bacteriostatic activity is achieved when antibacterial agents reduce <3 log_10_ cfu from the initial inoculum [22]. This study showed that APFD (MIC) and APFH (MIC) extracts reduced *S*. *mutans* by about >3 log_10_ cfu after 8 hours of incubation. Both extracts killed the bacteria after 8 hours of incubation. Leaf extracts (APLH and APLM) were shown to have fewer antibacterial activities compared to flowers. *A*. *paniculata* flowers have been used traditionally to treat toothaches more than *A. paniculata* leaves [23]. Traditionally, *A*. *paniculata* flowers were pounded to powder and then applied on tooth surface to reduce the pain. Investigation of phytochemicals is a crucial part of confirming the ethnomedicine values of certain parts of medicinal plants. This study was furthered to determine the phytochemicals of AP flower extracts since they were more potent and possessed greater antibacterial activity when compared to AP leaf extracts [17].

In phytochemical analysis, the major bioactive compounds of APFH and APFD extracts were fatty acids such as palmitic, oleic, linoleic, and linolenic acids which were also reported as major and common constituents in most plants [24]. APFH and APFD extracts contain all the major components of fatty acids, and the highest fatty acids were hexadecanoic and oleic acid. An earlier study found that hexadecanoic and oleic acids exhibited antibacterial properties against pathogens. Hexadecanoic acid (palmitic acid) is a saturated fatty acid, and its chemical formula is CH_3_(CH_2_)_14_COOH [25]. A previous study reported that hexadecanoic acid exhibited antibacterial activity against *Staphylococcus aureus*, *Pseudomonas aeruginosa*, and *Klebsiella pneumoniae* [26]. Shaaban et al. (2021) discovered that hexadecanoic acid was the main compound in clove alcoholic extract and possessed antibacterial activities against pathogen bacteria isolated from diabetic patients' swabs [27]. Compounds of oleic acid are monounsaturated fatty acids, and their chemical formula is C_18_H_34_O_2_ [24]. Agoramoorthy et al. reported that oleic acid exhibited antibacterial activities against Gram positive and Gram negative bacteria such as *Bacillus subtilis*, *Pseudomonas aeruginosa*, and *Escherichia coli* [28]. This compound also possessed antifungal activities against *Candida* spp. A previous study also reported that oleic acid inhibited bacterial growth of *Staphylococcus aureus* by disturbing the bacteria's enzyme for carrier protein (enoyl-acyl carrier protein reductase, FabI) [29]. The antibacterial activities of fatty acids such as hexadecanoic and oleic acid are stimulated by their structure, shapes, number of carbons, positions, and orientation of double bonds [30]. Fatty acid compounds disrupted bacterial membranes and inhibited fatty acid synthesis in microorganisms. Therefore, SEM and TEM analysis have been done to observe the morphological changes in *S*. *mutans* cell membrane treated with APFD and APFH extracts.

SEM and TEM analysis of treated *S*. *mutans* showed membrane cell damage and lysis due to cytoplasm leakage. A study by Parsons et al. (2012) reported that fatty acid was an antibacterial agent which depolarized the cells by creating pores in the membrane [31]. Linoleic acid has been previously shown to alter peptidoglycan synthesis in *S*. *aureus* [32]. Peptidoglycan is an essential component that builds the cell wall of bacteria. The changes in the outer membrane can be visualized by SEM and pinpoint the possibility of plasma membrane leakage and loss of cell functionality [33]. Meanwhile, TEM showed the structure of the plasma membrane, the roughness of the outer surface, and the irregularity of the subcellular structures. Fatty acid bioactive compounds modify the cell membrane, cytoplasm, enzymes, and proteins of the cells. Furthermore, fatty acids disrupted the microbial metabolism and caused leaking of ions, which led to cell death [34]. These analyses (SEM and TEM) confirmed that fatty acid in *A. paniculata* caused the abnormal cell morphology in *S. mutans*, possibly due to membrane leakage, ultimately resulting in cell lysis.

Transcriptomic profile analysis was done to investigate the gene regulation of *S. mutans* treated with *A. paniculata* extracts, especially in peptidoglycan synthesis. RNA sequencing is a new technology for transcriptome analysis profiling which can provide quantitative analysis of all transcripts with high accuracy and sensitivity [35]. Besides, RNA sequencing can expose specific biological functions affected after treatment with natural products or drugs [36]. Molecular analysis confirmed the results from SEM, TEM, and phytochemical analysis; that is, fatty acids disrupted the membrane cells of *S. mutans*. In this study, the genes for peptidoglycan biosynthesis were downregulated (Table 6) after *S*. *mutans* was exposed to APFD. These transcriptional changes are partially in agreement with the previous report using P. aeruginosa in which the drugs inhibited the murC and murD gene regulations. They also found that cell of P. aeruginosa was lysed in SEM analysis [37]. The downregulated genes were related to cell envelope biosynthesis in *S. mutans* exposed to APFD due to disruption of the electron transport and low production of ATP. ATP is a fundamental element for many metabolic processes in bacteria, including cell wall biosynthesis and protein synthesis [37]. *MurC* and *MurD* genes are involved in the accumulation of L- and D-amino acids to form UDP-MurNAc-L-Ala-*γ*-D-Glu-meso-A2pm-D-Ala-D-Ala of peptidoglycan [38]. The inhibition of both genes will disrupt the process of creating the peptidoglycan, which is sufficient to determine the cell shape [39].

The transcriptomic analysis showed that DNA replication genes of S. mutans were downregulated after treated with APFD. *dnaG* (primase) and *ssb* genes are hexameric helicase enzymes that act as the replicative DNA polymerase to process DNA synthesis [40]. DNA primase is a crucial molecule that produces RNA primers that are used to form Okazaki fragments (on DNA strands) [41]. The inhibition of primase genes (*dnaG* and *ssb*) is expected to halt DNA replication and inhibit cell proliferation [42]. Therefore, DNA primase is a potential gene for clinical targets for novel antibiotics. DNA replication inhibition has shown an effective antibacterial activity against bacterial pathogens. Kling et al. (2015) reported that peptide of griselimycin targeted DNA replication genes and caused *Mycobacterium tuberculosis* death [43]. Other than that, the inhibition of DNA replication genes stopped the growth of *S*. *aureus*. Inhibition of DNA replication will affect the growth of several bacteria [44]. Protein and DNA replication genes such as *ssb*, *dnaG*, *rnh3*, and *holB* have the potential to be an attractive drug discovery targets [42]. *Streptococcus mutans* is a common bacterium that initiates dental caries. The mechanism of action of APFD extracts was lysing the cell wall and inhibiting the DNA replication of *S. mutans*. This finding will reduce the incidents of dental caries worldwide.

## 5. Conclusions

In conclusion, *A*. *paniculata* extracts acted as bactericidal agents toward *S*. *mutans*. Bioactive compounds presented in the flower extracts such as oleic and hexadecenoic acids are the main constituents considered to be responsible for antibacterial activity. This study suggested that the mode of action of *A*. *paniculata* flower extracts was to disrupt the cell wall and inhibit the DNA replication of *S*. *mutans*.

## Figures and Tables

**Figure 1:** SEM analysis of *S*. *mutans* treated with APFH and APFD compared with untreated cells: (a) untreated *S*. *mutans*, (b) *S*. *mutans* treated with APFH (12.5 mg/mL), (c) *S*. *mutans* treated with APFH (50 mg/mL), (d) *S*. *mutans* treated with APFD (12.5 mg/mL), and (e) *S*. *mutans* treated with APFD (50 mg/mL). The morphology of untreated cell was aggregated (i); meanwhile, treated cells were elongated (ii), shrunk (iii), small (iv), and lysed (v).

**Figure 2:** TEM analysis of *S*. *mutans* treated with APFH and APFD compared with untreated cells: (a) untreated *S*. *mutans*, (b) *S*. *mutans* treated with APFH (12.5 mg/mL), (c) *S*. *mutans* treated with APFH (50 mg/mL), (d) *S*. *mutans* treated with APFD (12.5 mg/mL), and (e) *S*. *mutans* treated with APFD (50 mg/mL). Some characteristics of untreated bacteria were clearly seen such as granules, vacuoles and encapsulated structure (i); meanwhile, the cell wall of treated bacteria was lysed (ii) and distorted (iii) with formation of hollows (iv).

**Figure 3:** Total ion chromatogram of APFD extract. The highest peak for the APFD extract was linoelaidic acid (retention time: 39.46).

**Figure 4:** Total ion chromatogram of the APFH extract. The highest peak for the APFH extract was hexadecanoic acid (retention time: 34.63).

**Figure 5:** Total DEGs of *S*. *mutans* after treatment with APFD extract. Out of 1266 genes, 622 were downregulated and 644 were upregulated.

**Figure 6:** DEG analysis of *S*. *mutans* treated with APFD (MIC). (a) Heatmap clustering of all DEGs (1 < log_2_FC > 1 and *p* value < 0.05) in *S*. *mutans* treated with APFD. Each row represents one sample, and each column represents one gene. (b) Volcano image of gene regulation of *S*. *mutans* treated with APFD (MIC). Green color represents downregulated genes, and red color represents upregulated genes.

**Figure 7:** (a) Gene ontology category of DEGs in molecular function. The highest downregulated gene in molecular function was nucleic acid binding. (b) Gene ontology category of DEGs in cellular component (CC). Genes of cytoplasm were the highest downregulated genes in cellular component. (c) Gene ontology category of biology process (BP) showing downregulated genes in respective processes.

**Figure 8:** KEGG enrichment scatter plot of DEGs (downregulated). The *y*-axis shows the name of the pathway and the *x*-axis shows the rich factor. Dot size represents the number of different genes, and the color indicates the *q* value.

**Table 1:** Time-kill assessments of *A*. *paniculata* extracts against *S*. *mutans*.

Log_10_ cfu/mL					
Concentrations of extracts	0 h	4 h	8 h	24 h	28 h
Negative control	8.75	8.74	8.67	8.13	8.01
APLM: 100 mg/mL	8.75	0	0	0	0
APLM: 50 mg/mL	8.75	6.80	6.49	5.63	5.93
APLM: 25 mg/mL (MIC)	8.75	7.67	7.58	5.79	5.55
APLH: 100 mg/mL	8.75	5.52	0	0	0
APLH: 50 mg/mL	8.75	6.92	5.93	4.43	0.00
APLH: 25 mg/mL (MIC)	8.75	7.77	7.62	6.74	6.46
APFD: 50 mg/mL	8.75	6.39	6.09	0	0
APFD: 25 mg/mL	8.75	6.41	6.04	5.75	5.19
APFD: 12.5 mg/mL (MIC)	8.75	6.57	5.88	5.70	4.67
APFH: 50 mg/mL	8.75	5.19	0	0	0
APFH: 25 mg/mL	8.75	6.83	5.69	5.18	4.86
APFH: 12.5 mg/mL (MIC)	8.75	6.84	5.90	5.07	4.99

MIC values of APFH and APFD were reduced by more than 3 log_10_ cfu/mL of *S*. *mutans* when compared to MIC of leaf extracts (APLM and APLH).

**Table 2:** Phytochemicals identified in APFD extracts by GCMS analysis.

Retention time	Area (%)	Chemical name
17.3146	0.0169	Octanoic acid
36.6133	0.0412	n-Hexadecanoic acid
37.1087	0.1188	Oleic acid
37.4468	0.1086	Oleic acid
37.913	0.1672	12-Octadecenoic acid, methyl ester
38.187	0.2142	Phytol
39.3177	18.7013	9,12-Octadecadienoic acid (Z,Z)-
39.4226	6.3737	9,12-Octadecadienoic acid (Z,Z)-
39.466	6.9992	Linoelaidic acid
39.7141	5.0556	Octadecanoic acid
39.9297	1.2436	9,12-Octadecadienoic acid (Z,Z)-
44.785	0.1945	Linoelaidic acid
44.9365	1.6721	Hexadecanoic acid, 2-hydroxy-1-(hydroxymethyl)ethyl ester
45.2163	0.2291	9,12-Octadecadienoic acid (Z,Z)-
45.2921	0.0962	Linoelaidic acid
45.3854	0.2939	9,12-Octadecadienoic acid (Z,Z)-
45.5427	0.2693	9,12-Octadecadienoic acid (Z,Z)-
45.6185	0.0975	Linoelaidic acid
47.0932	0.0621	10,13-Octadecadienoic acid, methyl ester

Linoelaidic, octadecanoic, and palmitoleic acids were the major compounds in APFD extracts.

**Table 3:** Phytochemicals identified in APFH extracts by GCMS analysis.

Retention time	Area (%)	Chemical name
11.4918	1.307	Hexanoic acid
34.63	7.2589	Hexadecanoic acid, methyl ester
35.191	0.2576	Palmitoleic acid
35.6865	11.0542	n-Hexadecanoic acid
35.9896	1.3283	Eicosane (C20)
38.8689	6.1305	Oleic acid
43.048	1.7492	Acetamide, N-(2-phenylethyl)-
47.4836	0.9143	Eicosane

Hexadecanoic and oleic acids were the major compounds in the APFH extract.

**Table 4:** The concentration and RNA integrity number (RIN) of *S*. *mutans* treated with APFD and untreated bacteria (control).

Samples	Organism	Concentrations (ng/*µ*L)	RNA integrity number (RIN)	Total amount (*µ*g)
Control (1)	*S*. *mutans*	117.34	9.0	5.08
Control (2)	*S*. *mutans*	149.52	9.2	5.78
Treatment (APFD)	*S*. *mutans*	82.20	8.6	3.40
Treatment (APFD)	*S*. *mutans*	65.20	8.4	2.40

**Table 5:** Mapping analysis of the untreated and treated genome.

Sample name	Treated 1	Treated 2	Control 1	Control 2
Total reads	16016284	19238986	15934552	19460034
Total mapped reads	15305549	18469977	15447751	18883637
Uniquely mapped reads	14894816	17318063	15093404	18584375
Multiple mapped reads	410733	1151914	354347	299262
Total mapping rate	95.56%	96%	96.94%	97.04%
Unique mapping rate	93%	90.02%	94.72%	95.50%
Multiple mapping rate	2.56%	5.99%	2.22%	1.54%

SmuNN2025 genome was used as reference genome. The result of the mapping was more than 90% for all the samples.

**Table 6:** Log_2_ fold change of downregulated genes in APFD-treated *S*. *mutans*.

Gene name	Log_2_ fold change	*P* value	Gene description
*SmuNN2025_1359*	−1.6044657	2.09*E*−29	DNA polymerase III, delta subunit
*ssb*	−0.6788083	1.88*E*−14	Putative single-stranded DNA-binding protein
*dnaG*	−0.5734505	3.44*E*−11	DNA primase catalytic core, N-terminal domain
*rnh3*	−0.3960807	0.00051026	Putative ribonuclease PF01351: ribonuclease HII
*holB*	−0.3897243	0.00139286	Putative DNA polymerase III delta subunit
*murD*	−0.855528	1.69*E*−14	Putative D-glutamic acid adding enzyme
*uppS*	−1.1305843	1.94*E*−14	Putative undecaprenyl pyrophosphate synthetase
*murC2*	−0.7820073	1.92*E*−11	Putative UDP-N-acetylmuramyl tripeptide synthetase
*pbp2b*	−0.5783955	4.89*E*−09	Penicillin-binding protein dimerisation domain
*murE*	−0.4486175	3.23*E*−05	Putative UDP-N-acetylmuramoyl-L-alanine-D-glutamate-
*murN*	−0.403607	0.00089	Putative peptidoglycan branched peptide synthesis protein
*murB*	−0.440412	0.002353	Putative UDP-N-acetylenolpyruvoylglucosamine reductase

The genes were involved in biosynthesis peptidoglycan and DNA replication pathway (KEGG).

**Table 7:** Log_2_ fold change of upregulated genes in APFD-treated bacteria.

Gene name	Log_2_ fold change	*P* value	Gene description
*pdhD*	2.8355	1.30*E*−186	Putative dihydrolipoamide dehydrogenase
*pf1*	2.2289	2.37*E*−145	Pyruvate formate-lyase
*pdhA*	2.5844	2.45*E*−106	Putative pyruvate dehydrogenase E1 component alpha subunit
*SmuNN2025_1677*	2.0384	3.69*E*−63	Beta-lactamase superfamily domain
*glk*	1.1948	2.12*E*−34	Putative glucose kinase
ldh	0.9586	3.00*E*−33	Lactate dehydrogenase
*serA*	0.3443	0.0001	Putative D-3-phosphoglycerate dehydrogenase

All of the genes involved in microbial metabolism in diverse environments (KEGG pathway).

## Data Availability

The study data are available from the corresponding author on reasonable request. The whole methodology of this study is included in the Materials and Methods section.
